RETRACTED

# Maize *opaque10* Encodes a Cereal-Specific Protein That Is Essential for the Proper Distribution of Zeins in Endosperm Protein Bodies

**DOI:** 10.1371/journal.pgen.1006270

**Published:** 2016-08-19

**Authors:** Dongsheng Yao, Weiwei Qi, Xia Li, Qing Yang, Shumei Yan, Huiling Ling, Gang Wang, Guifeng Wang, Rentao Song

**Affiliations:** 1 Shanghai Key Laboratory of Bio-Energy Crops, School of Life Sciences, Shanghai University, Shanghai, China; 2 Coordinated Crop Biology Research Center (CBRC), Beijing, China; 3 National Maize Improvement Center of China, China Agricultural University, Beijing, China; University of Minnesota, UNITED STATES

## Abstract

Cereal storage proteins are major nitrogen sources for humans and livestock. Prolamins are the most abundant storage protein in most cereals. They are deposited into protein bodies (PBs) in seed endosperm. The inner structure and the storage mechanism for prolamin PBs is poorly understood. Maize *opaque10* (*o10*) is a classic opaque endosperm mutant with misshapen PBs. Through positional cloning, we found that *O10* encodes a novel cereal-specific PB protein. Its middle domain contains a seven-repeat sequence that is responsible for its dimerization. Its C terminus contains a transmembrane motif that is required for its ER localization and PB deposition. A cellular fractionation assay indicated that O10 is initially synthesized in the cytoplasm and then anchored to the ER and eventually deposited in the PB. O10 can interact with 19-kD and 22-kD α-zeins and 16-kD and 50-kD γ-zeins through its N-terminal domain. An immunolocalization assay indicated that O10 co-localizes with 16-kD γ-zein and 22-kD α-zein in PBs, forming a ring-shaped structure at the interface between the α-zein-rich core and the γ-zein-rich peripheral region. The loss of O10 function disrupts this ring-shaped distribution of 22-kD and 16-kD zeins, resulting in misshapen PBs. These results showed that O10, as a newly evolved PB protein, is essential for the ring-shaped distribution of 22-kD and 16-kD zeins and controls PB morphology in maize endosperm.

## Author Summary

Through the positional cloning of the maize classic endosperm mutant *opaque10* (*o10*), we identified a novel protein critical for PB morphology. *O10* is a fast-evolving cereal-specific gene with recent origin. A thorough characterization of its three functional domains revealed its important functions for storage protein deposition and organization in PBs. O10 determines a ring-shaped layer in PBs through direct interaction with two major storage proteins (22-kD and 16-kD zeins). This newly characterized PB layer maintains a stable spherical morphology for PB. This study advanced our understanding of PB structure and function. Furthermore, this study demonstrated the origin of a new functional gene and the functional evolution of a storage organelle that is highly valuable to humans.

RETRACTED

## Introduction

Cereal crops are major source of the world’s food supply [1,2]. Many storage proteins in cereal grains are valuable nitrogen sources for humans and livestock [3]. Prolamins are major storage proteins that occur only in cereal grain endosperm [4]. Studies of the protein storage mechanism are critical for improving cereal grain nutritional quality. However, the exact storage mechanisms of prolamins remain poorly understood.

Maize (*Zea mays*) is the first staple cereal crop in the world. Maize kernels primarily contain 70–75% starch, 8–10% protein, and 4–5% lipids [5]. More than 60% of proteins are prolamins and are also known as zeins. Zeins are divided into four major classes, namely α-zeins (19 and 22 kD), β-zein (15 kD), γ-zeins (16, 27, and 50 kD), and δ-zeins (10 and 18 kD) according to their primary structure and different solubilities. α-Zeins are encoded by a multigene family, and other zeins are encoded by single-copy genes [6–8]. Zeins are synthesized in endosperm cells [9] by membrane-bound polyribosomes, transported into the lumen of the rough endoplasmic reticulum (RER) and then aggregated into the formation of protein body (PB) [10,11].

The exact process of zein deposition into PB remains unclear. However, the immunolocalization of different zeins showed that they have a specific localization during the PB packing process [12]. Initially, only β- and γ-zein proteins accumulate in the PBs, and then α- and δ-zeins penetrate into the matrix formed by β- and γ-zeins and expand the PBs into larger spherical structures. The β- and γ-zeins then become a thin layer that surrounds the PBs [12,13]. The 19-kD α-zein is located throughout the PB core, but the 22-kD α-zein is located only in a discrete ring at the interface between the α-zein-rich core and the 27-kD γ-zein-rich peripheral region [14]. However, the mechanism that underlies distinct zein distribution patterns remains poorly understood.

Studies of opaque endosperm mutants shed light on the development of PBs. The first class of opaque mutants reduced the zein content, resulting in small, unexpanded PBs, such as *opaque2* (*o2)*, *o6*, *o7*, and *mto14*0 [15–18]. The second class of opaque mutants, such as *floury2* (*fl2*), *fl4*, *De-B30* and *Mc*, has phenotypes that are derived from defective zeins [19–22]. The third class of opaque mutants, such as *floury1* (*fl1*) and *o1*, does not cause qualitative or quantitative changes in the zeins. *fl1* encodes a PB membrane protein that affects the distribution of 22-kD α-zein in the PBs. In *fl1*, the 22-kD α-zein is dispersed more randomly throughout the PBs [14]. *o1* encodes a plant-specific myosin protein that is responsible for ER morphology and motility, therefore forming smaller but more PBs in the endosperm [23]. These studies indicate that the perfect packing of zeins in PBs depends on not only zeins but also other proteins, but thus far, only a few have been studied.

RETRACTED

In this study, we cloned and studied *opaque10 (o10)*, a new opaque mutant that affects zein assembly and PB morphology. *O10* encodes a new protein that is only present in cereal plants. O10 has unique sequence features that are responsible for its unique sub-cellular distribution and accumulation. O10 directly interacts with zein proteins and is required for the ring-shaped distribution of 22-kD and 16-kD zeins in PBs in particular. The cloning of *O10* expanded our understanding of the mechanism of proper zeins distribution within PBs and its relations to PB shape and endosperm opacity.

## Results

### Maize *o10* produces misshapen PBs

*o10* is a putative ethylmethane sulfonate (EMS)-induced mutant that was generated by M.G. Neuffer and named by Oliver Nelson [24]. The *o10-N1356* mutant from the Maize Genetics Cooperation Stock Center was crossed into the W22 genetic background. On the F2 ears, the progenies exhibit a 3:1 segregation of wild-type (+/+ and *o10*/+) (vitreous) and opaque (*o10*/*o10*) kernel phenotypes, indicating that *o10* corresponded to a single recessive gene mutation.

The *o10* kernels exhibited a typical opaque endosperm phenotype when viewed on a light box. The transverse section of the mature kernels showed a much thinner layer of vitreous endosperm than that of the wild-type (Fig 1A). A scanning electron microscopy (SEM) examination of the mature kernel endosperm showed that the starch granules in the peripheral region of the mutant kernels were loosely packed (S1A Fig).

**Fig 1:** Map-based cloning and identification of *O10*. (A) Light transmission and transverse sections of the wild-type (WT) and *o10* kernels from the same F2 ear. Bars = 1 cm. (B) Observation of PBs in the wild-type and *o10* developing kernels at 21 DAP by TEM. Bars = 1 μm. PB, protein body; SG, starch granules. (C) The *o10* locus was mapped to a 110-kb region on chromosome 1 with five candidate genes. (D) Structure and mutation site of the *O10* gene. The lines represent introns, and the black boxes represent exons. (E) Schematic diagram of the maize O10 and o10 protein structures. aa, amino acid. (F) Immunoblot comparing the accumulation of O10 in the wild-type and *o10* mature kernels. Anti-tubulin was used as a sample loading control.

RETRACTED

To examine if there was a corresponding change in the storage components of the mutant kernels, we examined the major biochemical components in the mutant and wild-type kernels. A quantitative analysis showed that there was no distinct change in the zein, non-zein, and total proteins in opaque kernel endosperm compared the wild-type (S1D Fig). The results of the SDS-PAGE also indicated that there was no obvious difference in the major zein components between the mutant and wild-type endosperm at either the mature or developing stages (S1C Fig). We also analyzed the total starch and lipid contents but did not find obvious differences between the *o10* and wild-type kernels (S1E and S1F Fig).

The endosperm resin section at 12 d after pollination (DAP) and 18 DAP showed that the starch granule development was not affected in *o10* (S1B Fig). Transmission electron microscopy (TEM) revealed that PBs were spherical in the wild-type endosperm, whereas many PBs were irregularly shaped in the *o10* endosperm (Fig 1B). Based on these results, O10 might function in PB formation.

### Map-based cloning of *O10*

We used a map-based approach to clone *O10*. After characterizing a population of approximately 12,000 opaque mutant kernels and 1,500 wild-type kernels from the F2 population, the *o10* gene was placed between the molecular markers SSR217401-a and Indel557-1, which is a region that encompasses a physical distance of 110 kb. This region was covered by 2 BAC clones (AC204586 and AC217401). There are five candidate genes within the interval (Gene 1: AC217401.3_FG004, Gene 2: GRMZM2G510280, Gene 3: GRMZM2G346263, Gene 4: GRMZM2G510235 and Gene 5: GRMZM2G044557) (Fig 1C). Sequence comparison of the five candidate genes between wild-type and mutant alleles revealed a typical EMS-induced G/A transition at the 3’ end of intron 6 in Gene 3 (Fig 1D). This point mutation resulted in the retention of a 95-bp intron (intron 6), causing a frame-shift and a premature stop codon in the mature transcript.

To confirm that Gene 3 is the *O10* gene, functional complementation was performed using a transformed wild-type candidate gene allele. Phenotyping and genotyping analysis indicated the transgenic kernels carrying the transformed wild-type Gene 3 sequence functionally complemented the lost function of *o10* and rescued the mutant phenotype (S2A–S2C Fig). We also made an RNAi construct to target the Gene 3 sequence for maize transformation. Phenotyping and genotyping analysis indicated that all the transgenic kernels exhibited an opaque phenotype (S2D–S2F Fig). These results indicated that Gene 3 is the *O10* gene.

RETRACTED

*O10* encodes a protein with 1,059 amino acids, but in *o10*, it encodes 1,009 amino acids, with the first 963 amino acids being identical to those of the wild-type protein (Fig 1E). In using the antibody (anti-O10) that was raised against the N-terminal (1–541 aa) region of this protein, a protein with an apparent molecular weight of approximately 220 kD was detected in all the wild-type and *o10* mature kernels; however, the protein contents of the *o10* kernels dramatically decreased compared to those of the wild-type. In using the antibody (anti-O10-C) that was raised against the C-terminal (1020–1059 aa) region of the protein, the protein was detected in the wild-type mature kernels but not in mutant mature kernels (Fig 1F).

### *O10* encodes a novel cereal-specific protein

NCBI BLAST searches using the full-length O10 revealed that O10 is a novel protein that is only present in cereal species (Fig 2A). The N-terminal portion (1–268 aa) of O10 has a homologous sequence in different plants. Most of these plants are dicotyledons, such as *Glycine max* and *Nicotiana tomentosiformis*, but surprisingly not *Arabidopsis* (Fig 2A). In the middle portion, O10 has a repeating region containing seven unknown repeats (269–786 aa). The homologous sequences of these repeats are only present in cereal species. However, the repeat number in different cereals is highly variable. In maize, the repeat number is seven (*Zea mays*-1 to *Zea mays*-7), and in sorghum, the number is two (*Sorghum bicolor*-1 and *Sorghum bicolor*-2). In other cereal species, only one repeat is found (S3A Fig). O10 has a predicted transmembrane domain in its C terminus (1002–1024 aa). The transmembrane domain in the C terminus is highly conserved among cereal species. It is also sporadically present in plants (*Nelumbo nucifera*), insects (*Bactrocera cucurbitae*) and even in bacteria (*Chryseobacterium palustre*) (S3B Fig).

**Fig 2:** Phylogenetic analyses of O10 and the expression pattern of *O10*. (A) The O10 protein and currently identified homologous of O10 from NCBI were aligned by ClustalW. The phylogenetic tree was constructed using MEGA 6.0. Distances were estimated with a neighbor-joining algorithm, and bootstrap support is indicated to the left of branches. *Selaginella moellendorffii* homologous protein was used as an outgroup. The different general structural classes of O10 and its homologous proteins are shown on the right and below the tree. (B) RNA expression level of *O10* in various tissues. Ubiquitin was used as an internal control. For each RNA sample, three technical replicates were performed. Representative results from two biological replicates are shown. Error bars represent SD. Transcript abundance is indicated relative to the husk. (C) Immunoblot analysis of O10 accumulation in various tissues. Anti-tubulin was used as a sample loading control. (D) Expression profiles of *O10* during maize kernel development. Ubiquitin was used as an internal control. For each RNA sample, three technical replicates were performed. Representative results from two biological replicates are shown. Error bars represent SD. Transcript abundance is indicated relative to 35 DAP. (E) Immunoblot analysis of O10 accumulation during maize kernel development. Anti-tubulin was used as a sample loading control.

RETRACTED

### *O10* is preferentially expressed in the developing kernel

A real-time quantitative PCR analysis was used to examine *O10* gene expression in different tissues. The results indicated that *O10* is most significantly expressed in immature kernels; however, lower levels of expression were also detected in other tested tissues (Fig 2B). An immunoblot analysis with an O10-specific antibody (anti-O10) showed that the O10 protein significantly accumulated in the kernel but was barely detected in the tassel, ear, silk, leaf and sheath (Fig 2C). In developing kernels, *O10* expression was clearly detected at 7 DAP and sharply increased and peaked at approximately 11 DAP. The expression then gradually decreased until 35 DAP, with a second peak at approximately 23 DAP (Fig 2D). The O10 protein was only detectable at 11 DAP by an O10-specific antibody (anti-O10) and then gradually increased during kernel development and continuously accumulated until the late development stage (35 DAP) (Fig 2E). In mature kernels, the O10 protein also highly accumulated. This result indicated that the O10 protein continuously accumulated during kernel development.

### Seven-repeat domain of O10 is responsible for its dimerization

In using the antibodies (anti-O10 and anti-O10-C), the apparent size of the detected protein was approximately twice that of the predicted one (114.58 kD, http://www.expasy.org/tools/pi_tool.html). Gel filtration chromatography also indicated that O10 was primarily detected in fraction 4, which is larger than 158 kD (fraction 5) (S4A Fig). The full-length ORF of *O10* expressed in *E*. *coli* also showed a similar apparent size (Fig 3A and 3B). We speculated that the O10 protein likely presented as a dimer; however, dimerization likely did not occur through a di-sulfide bond between cysteines because strong denaturing treatment did not disrupt the dimer (S4B Fig). The full-length of O10 ORF was further divided into three fragments and expressed in *E*. *coli* (Fig 3A). Only the induced protein of the second fragment containing the seven-repeat portion still displayed an increased apparent size, which was approximately twice the predicted size (Fig 3B). Therefore, the seven-repeat sequence in the middle portion of O10 was responsible for forming a potential dimer. Previous studies indicated that the resistance of the dimer to denaturant is common to several proteins that form hydrophobic intermolecular interactions [25,26]. Thus, we analyzed the hydrophobicity of the seven-repeat domain of O10 and found that every repeat had a hydrophobic segment. We postulated that the dimer of O10 might be formed by the intermolecular hydrophobic forces of the seven-repeat domain (S5 Fig).

RETRACTED

**Fig 3:** Expression of O10-derived fragments in *E*. *coli* cells. (A) Schematic representations of O10-derived fragments used in the expression in *E*. *coli*. 1, residues 1–268 aa; 2, residues 269–786 aa; 3, residues 787–1059 aa; and 4, the full length ORF of O10. Their molecular weights (MW) were predicted by ExPASy. (B) SDS-PAGE gel of the expressed proteins stained with Coomassie blue. We used 15 μg of total *E*. *coli* cell protein per lane. Red arrowheads note the expressed protein of O10-derived fragments in each lane.

### The *o10* mutation affects the distribution and accumulation of O10 in the kernel

Gene cloning and sequence analysis indicated that the *o10* mutation led to the loss of the C-terminal O10 transmembrane domain, which might have a sub-cellular membrane-localization function. The ORFs corresponding to wild-type *O10* and mutated *o10* were fused to the C terminus of YFP to produce the YFP-O10 and YFP-o10 constructs, respectively. These constructs were used to agroinfiltrate *N*. *benthamiana* leaves. A confocal microscope observation showed that YFP-O10 fluorescence was primarily presented by some unknown spherical vesicles (Fig 4A). We co-expressed YFP-O10 with an ER marker (mCherry-HDEL) in *N*. *benthamiana* leaves, and the results showed that these unknown spherical vesicles could co-localize with the ER around the nucleus (Fig 4B). However, these spherical vesicles were not observed in the YFP-o10 agroinfiltrated cells (Fig 4C). YFP-o10 could co-localize with ER throughout the cells (Fig 4D). These results indicated that the transmembrane domain was responsible for the localization of O10 in *N*. *benthamiana* cells.

**Fig 4:** The distribution and accumulation of O10 in the wild-type and *o10* developing kernels. (A) The subcellular localization of YFP-O10 fusion protein in *N*. *benthamiana* leaves. Bars = 20 μm. (B) O10 could co-localize with ER around the nucleus. Confocal microscopic images were taken from *N*. *benthamiana* leaves in which YFP-O10 and the ER maker (mCherry-HDEL) were co-expressed. Bars = 20 μm. (C) The subcellular localization of YFP-o10 fusion protein in *N*. *benthamiana leaves*. Bars = 20 μm. (D) o10 could co-localize with ER throughout the cells. Confocal microscopic images were taken from *N*. *benthamiana* leaves in which YFP-o10 and the ER maker (mCherry-HDEL) were co-expressed. Bars = 20 μm. (E) Immunoblot comparing accumulation of O10 in the wild-type and *o10* developing kernels. Anti-tubulin was used as a sample loading control. (F) Immunoblot analysis of O10 in the wild-type and *o10* cytoplasm fractions with anti-O10 antibody (50 μg of protein per lane). (G) Immunoblot analysis of O10 in the wild-type and *o10* total membrane fractions with anti-O10 antibody. Anti-BIP was used as a sample loading control. (H) Immunoblot analysis of O10 in the ER and PB fractions from the wild-type and *o10* developing kernel cells (21 DAP) with anti-O10 antibody. Anti-BIP was used as an ER marker, and Anti-22-kd α-zein was used as a PB marker.

RETRACTED

To explore the effects of the *o10* mutation in maize kernels, we first compared the gene expression of *O10* in the wild-type and mutant by real-time quantitative PCR. The wild-type and mutant kernels at three developmental stages (15 DAP, 18 DAP and 21 DAP) were analyzed. The results indicated that at the transcript level, *O10* expression exhibited no obvious differences between the wild-type and mutant (S6 Fig). We then used an immunoblot with an O10-specific antibody (anti-O10) to examine the O10 protein levels in the wild-type and mutant. Compared to the O10 in the wild-type, the o10 in the mutant kernels had similar protein accumulation levels at 15 DAP and 18 DAP. However, o10 dramatically decreased at 21 DAP in the mutant (Fig 4E). A similarly low level of o10 was also found in the mature kernels of the mutant (Fig 1F). Therefore, the mutation in *o10* does not affect its gene transcription but greatly affects its protein accumulation during kernel development.

We then used a cellular fractionation assay to detect the O10 distribution in the subcellular fractions during kernel development. The total proteins extracted from developing kernels of wild-type and *o10* at 15 DAP, 18 DAP and 21 DAP were then separated into soluble and total membrane fractions, respectively. An immunoblot analysis was performed with the O10-specific antibody (anti-O10). Both O10 and o10 had significant protein levels in the soluble (cytoplasmic) fractions, and no difference was found between wild-type and mutant kernels at 15 DAP, 18 DAP and 21 DAP (Fig 4F). However, in terms of total membrane fractions, o10 dramatically decreased in the mutant kernels in compared to the wild-type (Fig 4G). This result indicated that the mutation in *o10* greatly affected the partitioning and accumulation of o10 in the total membrane fraction.

RETRACTED

We further isolated the ER and PB fractions from the total protein of 21-DAP wild-type and *o10* kernels by discontinuous Suc gradient centrifugation. An immunoblot analysis indicated that there was an extremely high level of O10 accumulation in the wild-type within the PB fraction. However, in *o10*, there was a low level of o10 accumulation in both the ER and PB fractions (Fig 4H). These results indicated that in endosperm, O10 was predominantly deposited into PBs, and the mutation in *o10* greatly affected the deposition of o10 into PBs.

### O10 is deposited inside PBs and interacts with different zeins

The cellular fractionation assay found O10 to be predominantly deposited into PB fractions. Because PBs are surrounded by the ER, the O10 protein may be attached to the ER or may be located inside the PBs. We then purified the PBs of 21-DAP wild-type kernels and used Triton X-100 to peel off the ER surrounding the PB core and then analyzed the peel fraction (the surrounding ER) and the zein-rich interior PB core by immunoblot. Like 22-kD α-zein, the immunoblot results using anti-O10 antibody indicated that O10 primarily accumulated inside the PBs, with a much lower amount in the surrounding ER fraction (Fig 5A). This indicated that O10 is finally deposited inside the PBs. The immunoblot using an anti-O10-C antibody also detected a similar distribution of O10 in the PBs and surrounding ER (Fig 5A). This indicated that the TMD was still present in the O10 protein when it was deposited into the PB. To confirm the interior localization of O10 in PBs, an immunolocalization analysis was performed with an anti-O10 antibody (anti-O10) on ultrathin sections of 21-DAP wild-type kernels. The results indicated that O10 is indeed localized inside PBs. Moreover, we also observed a featured distribution of O10 in PBs at the interface between the 19-kD α-zein-rich region (the inner darker region) and the γ-zein-rich region (the peripheral lighter region) (Fig 5B).

**Fig 5:** Localization of O10 in the PB and the Interactions between O10 and different type of zeins. (A) Immunoblotting of O10 in the fraction of PB that was treated with Triton X-100. S, supernatant (the surrounding ER); P, pellet (the PB core). The fraction without Triton X-100 treatment was used as a negative control. Fractions were subjected to immunoblot analysis with antibodies against the N terminus of O10 (anti-O10), the C terminus of O10 (anti-O10-C), BIP (ER marker), or 22-kD α-zein (PB marker). (B) Immunolocalization of O10 in wild-type endosperm samples (21 DAP). The red arrowheads indicate O10 gold labeling on the PB; Bars = 0.5 μm. (C) O10-N represents the N terminus of O10 from 1–268 aa. The interaction between T-antigen and Human P53 was used as a positive control. The interaction between pGBKT7-O10-N and pGADT7-empty was used as a negative control. AD, activating domain; BD, binding domain. (D) LCI assay showing that the N terminus of O10 interacts with different types of zeins. Fluorescence signal intensities represent their interaction activities.

RETRACTED

The specialized localization of O10 in PBs suggested its potential function in association with zeins. A protein-protein interaction assay then was performed between O10 and different zeins with a yeast two-hybrid system. A full-length ORF (O10-full) and its three fragments, including the N terminus of O10 (O10-N, 1–268 aa), the middle region comprising the repeats (O10-M, 269–786 aa) and the C-terminal region (O10-C, 787–1000 aa), were inserted into pGBKT7 as baits. The O10-full, O10-M and O10-C baits all exhibited self-activation in yeast and were not suitable for further analysis. Only O10-N passed the self-activation test and was used for the interaction assay.

The coding sequences 19-kD α-zein (AF546188.1), 22-kD α-zein (GRMZM2G044625), 15-kD β-zein (GRMZM2G086294), 16-kD γ-zein (GRMZM2G060429), 27-kD γ-zein (GRMZM2G138727), 50-kD γ-zein (GRMZM2G138689), and 10-kD δ-zein without the signal peptide were inserted into pGADT7 as the preys. Yeast strain AH109 was co-transformed with pGBKT7-bait and pGADT7-preys. Matings containing both the bait and prey were spotted on SD/-Leu/-Trp medium and SD/-Ade/-His/-Leu/-Trp medium as a series of dilutions. All of the matings had similar numbers of vigorously growing colonies on SD/-Leu/-Trp media. However, only the matings between the O10-N and 19-kD α-zein, 22-kD α-zein, 16-kD γ-zein and 50-kD γ-zein prey constructs could grow on SD/-Ade/-His/-Leu/-Trp medium, while the other mating combinations could not grow. This result implied that the N-terminal portion of O10 probably had protein-protein interactions with 19-kD α-zein, 22-kD α-zein, 16-kD γ-zein and 50-kD γ-zein (Fig 5C). To verify the interaction between O10 and different zeins, we performed a luciferase complementation image (LCI) assay. The N terminus of O10 (O10-N) was fused to the N-terminal domain of luciferase (NLUC), and the full-length of 19-kD α-zein, 22-kD α-zein, 15-kD β-zein, 16-kD γ-zein, 27-kD γ-zein, 50-kD γ-zein, and 10-kD δ-zein without the signal peptide were separately fused to the C-terminal domain of luciferase (CLUC). The results showed that the co-transfection of O10-N-NLUC with 19-kD α-zein-CLUC, 22-kD α-zein-CLUC, 16-kD γ-zein-CLUC or 50-kD γ-zein-CLUC could produce strong luciferase activity (Fig 5D), indicating that O10 can interact with these types of zeins in tobacco cells. These results confirmed the interaction of O10 with 19-kD α-zein, 22-kD α-zein, 16-kD γ-zein and 50-kD γ-zein.

RETRACTED

### *o10* PBs display abnormal 16-kD γ-zein and 22-kD α-zein localization

Considering that O10 can interact with 19-kD and 22-kD α-zeins and 16-kD and 50-kD γ-zeins, an immunolocalization analysis was performed for these zeins, as well as for the 27-kD γ-zein. In 21-DAP wild-type endosperms, the 19-kD α-zein, 22-kD α-zein, 27-kD γ-zein and 50-kD γ-zein all showed distinct distributions in the PBs, in agreement with previous studies [14,27]. The 16-kD γ-zein had a similar location as that of the 22-kD α-zein, which was at the interface between the β- and γ-zein-rich peripheral layer and the α-zein-rich inner region. In 21-DAP *o10* endosperm, the distribution of 19-kD, 27-kD and 50-kD zeins in PBs was the same as that in the wild-type. However, the 16-kD γ-zein and 22-kD α-zein changed in terms of their distinct distribution. The 16-kD γ-zein was diffused into the β- and γ-zein-rich peripheral layer, and they were no longer restricted to the interface layer. The 22-kD α-zein was also no longer restricted to the interface layer, but they diffused into the α-zein-rich core zone of PBs (Fig 6A). We merged ten immunolocalization pictures of 16-kD γ-zein, 22-kD α-zein and O10 into the same PB (Fig 6B).

**Fig 6:** The distribution of different types of zeins in wild-type and *o10* PBs. (A) Immunolocalization of O10, 16-kD γ-zein, 19-kD α-zein, 22-kd α-zein, 27-kD γ-zein and 50-kD γ-zein in the PBs of wild-type and *o10* at 21 DAP. Bars = 0.5 μm. (B) Ten pictures of each 16-kD γ-zein (blue dot), 22-kD α-zein (green dot) and O10 (red dot) were merged together in the same PB of wild-type and *o10* according to the distance from the protein body surface to the center of the gold particle, which was measured using ImageJ.

A real-time quantitative PCR analysis indicated that the expressions of 19-kD α-zein, 22-kD α-zein, 15-kD β-zein, 16-kD γ-zein, 27-kD γ-zein, 50-kD γ-zein, and 10-kD δ-zein at 18 DAP were similar between the wild-type and *o10*. At 24 DAP, most of the zeins still had similar expression levels; however, the 16-kD γ-zein had a significantly increased transcript level compared to that of the wild-type (S7 Fig). A more sensitive HPLC profiling analysis confirmed that the 16-kD γ-zein was the only significantly increased zein in mature *o10* kernels compared to the wild-type (S8 Fig). Therefore, *o10* not only changed the distribution of 16-kD γ-zein in PBs but also increased its accumulation in PBs.

RETRACTED

### The relationship of *o10* with other opaque mutants

Previous studies have shown that O1 and FL1 are two non-zein proteins that are directly related to PB development [14,23]. To test whether O10, O1 and Fl1 had direct interactions, a yeast two-hybrid assay of O10-N (1 aa-268 aa) with an O1-tail (877 aa-1520 aa) and full-length FL1 was performed. The results indicated that the N terminus of O10 could not interact with either O1-tail or FL1 in yeast (Fig 7A). The interaction between O10 and O1 or FL1 was further analyzed by an LCI assay. The full-length of O10 was fused to the C-terminal domain of luciferase (CLUC), and the C terminus of O1 (877–1520 aa) or FL1 (150–302 aa) was fused to the N-terminal domain of luciferase (NLUC). The results showed that the co-transfection of FL1-C-NLUC with O10-CLUC could produce strong luciferase activity (Fig 7B), while the co-transfection of O1-C-NLUC with O10-CLUC could not produce luciferase activity. These results indicated that O10 can interact with the C terminus of FL1 in tobacco cells.

**Fig 7:** The interactions of O10 with O1, HIP and FL1 and the accumulation of O10 in other opaque mutants. (A) Yeast two-hybrid interactions between the O10-N and O1-Tail, HIP and FL1. The interaction between T-antigen and Human P53 was used as a positive control. The interaction between pGBKT7-O10-N and pGADT7-empty was used as a negative control. AD, activating domain; BD, binding domain. (B) LCI showing that O10 interacts with HIP and FL1. Fluorescence signal intensities represent the interaction activities. (C) Immunoblot analysis of O10 and the accumulation of different zein proteins in different opaque mutants and corresponding wild-type mature kernels. Anti-tubulin was used as a sample loading control.

A previous study indicated that O1 interacts with an hsp70-interacting protein (HIP, GRMZM2G023275) [23]. We further tested whether HIP interacted with O10 by a yeast two-hybrid assay. The result indicated that O10-N might interact with HIP (Fig 7A). To verify the interaction between O10-N and HIP, we performed an LCI assay. The results showed that the co-transfection of O10-N-NLUC with HIP-CLUC could produce strong luciferase activity (Fig 7B). These results indicated that O10 may interact with HIP and FL1.

We also analyzed the accumulation of O10 and some types of zeins in other opaque mutants, including *o1*, *fl1*, *fl4*, *o2* and *o7*. The immunoblot results showed that in *o1*, *fl4* and *fl1*, there was no distinct change in the zein proteins compared to the wild-type, and the O10 content was decreased in *o1*, *fl4* but not in *fl1*. In *o2*, the contents of α-zeins and 50-kD γ-zein dramatically decreased; the O10 content did not change. In *o7*, the content of all zeins decreased, especially that of 16-kD γ-zein and 19-kD α-zein, and the O10 content dramatically decreased (Fig 7C).

RETRACTED

## Discussion

### *O10* encodes a fast-evolving cereal-specific protein

Newly created genes are common in many species. Distinct molecular processes contribute to the formation of new genes through processes such as gene duplication, gene fusion, or the alteration of the existing gene structure, or genes can arise from previously non-coding DNA [28]. For example, *Jingwei* (*Jgw*) is a recently evolved gene in *Drosophila* that encodes a protein containing two domains from two different proteins. Its chimeric structure is derived from exon shuffling between the *Adh* and *Ymp* genes, and it thereby acquired new biochemical functions [29,30]. The high rate of this chimeric gene origination is common in plants. In rice, 380 chimeric genes are recruited from previously existing genes [31]. A BLAST sequence analysis indicated that O10 is a cereal-specific protein. The N terminus of O10 has homologs in most plants (Fig 2). However, the TMD of the C terminus is rarely present in other plants, but it does exist in some insects and bacteria (S3 Fig). The middle portion of O10 with repeated regions only exists in the cereal family (Fig 2). Apparently, O10 is generated by the fusion of at least three distinct domains with independent origins. These sections were merged into one protein in cereals, most likely by similar gene fusion or shuffling mechanisms. Our results showed that the newly generated O10 protein has new biological functions that arise through a combination of different functional domains with different origins. O10’s new function is important for the development of PB in cereals; hence, such a random sequence fusion event might be functionally selected and inherited over the course of evolution. Furthermore, *O10* is still a fast-evolving gene. This statement is evidenced by the highly variable repeat number of the middle portion among O10 homologous proteins in different cereals (S3 Fig). Because O10 has an important function in PBs and is still subjected to fast evolution, we predict that the PBs in cereal endosperm might have a relatively recent origin and are still undergoing rapid evolution.

### O10 is a newly identified non-zein PB protein

Maize endosperm PBs consist mostly of zeins but also non-zein proteins. PBs can be induced in *Nicotiana benthamiana* leaves by transient transformations with Zera that are fused to a fluorescent marker protein (DsRed). The proteome analysis of these induced PBs revealed 195 additional proteins in addition to Zera-DsRed, including a broad range of proteins [32]. It is reasonable to predict that maize PBs would also have many non-zein proteins that participate in the formation of PB. Three non-zein proteins were characterized in maize PB, namely BIP (ER lumen binding protein), O1 and FL1. BIP is an ER chaperone and is associated with the folding and assembly of zeins in PB [33]. O1 encodes a plant-specific myosin protein that targets ER and PB. O1 is responsible for ER morphology and motility and affects the formation of PBs on the ER [23]. FL1 is an ER membrane-localized protein and can interact with 19-kD α-zein and 22-kD α-zein. This protein controls the proper distribution of 22-kD α-zein in PBs [14]. In this study, O10 was identified as a new non-zein protein in maize PB.

RETRACTED

Our results indicated that O10 was initially synthesized in the cytoplasm and was ultimately deposited inside the PBs. To be deposited inside the PBs, O10 should undergo at least three processes as follows: transport into the ER lumen, retention in the ER lumen, and deposition into PB. A sequence analysis indicated that O10 has no predicted signal peptide; thus, there may be other factors to aid O10 in entering the ER lumen across membranes. We found that the N terminus of O10 can interact with HIP (Fig 7). HIP is a cytosolic protein that interacts with the ATPase domain of HSP70 [34,35]. Genetic and biochemical evidence supports a role for cytosolic HSP70s in the post-translational translocation of precursor proteins into the ER and mitochondria [36,37]. Therefore, chaperone HSP70 might take part in the transportation of O10 into the ER lumen.

Many mechanisms can lead to protein retention in the ER lumen. The HDEL or KDEL tetrapeptides at the C terminus were identified as a retention signal in the ER for ER luminal proteins, such as in BIP [38,39]. The double-lysine motif (KKXX or KXKXX) in the C terminus of type I integral ER membrane proteins, such as Wbp1 in yeast, was identified as another ER retention signal [40]. The TMD was also shown to take part in protein retention in the ER lumen [41–43]. The *o10* mutation caused the loss of the TMD in the C terminus of O10 (Fig 1). The accumulation of o10 in the ER dramatically decreased when the TMD was absent (Fig 4). These results showed that the TMD in the C terminus of O10 plays an important role in O10 retention in the ER lumen. The suppressed ER function might directly affect the targeting and transportation of O10 to PB. In fact, in opaque mutants with disrupted ER functions, such as *o1* and *fl4*, the accumulation of O10 also significantly decreased (Fig 7).

An interaction with zeins would be consistent with the deposition of O10 inside the PBs. Among O10-interacting zeins, the 16-kD γ-zein appeared to be more important for O10 aggregation. There was a correlation between the accumulation of O10 and 16-kD γ-zein in other opaque mutants. In *fl1*, the contents of different zeins were barely affected, and the O10 content did not change. In *o2*, the contents of α-zeins and 50-kD γ-zein dramatically decreased; however, the O10 content did not change, as for the 16-kD γ-zein. In *o7*, all of the zeins were generally down-regulated, especially 16-kD γ-zein and 19-kD α-zein, and the O10 content dramatically decreased. Coincidentally, the expression and accumulation of the 16-kD γ-zein gene increased in o10, but the other zeins did not change (S7 and S8 Figs). The increased expression and accumulation of 16-kD γ-zein might be feedback regulation related to the failure of O10 deposition inside PBs together with 16-kD γ-zein.

RETRACTED

We proposed a possible model for the cellular route of O10 (Fig 8). O10 is initially synthesized in the cytoplasm and, perhaps with the aid of HIP and HSP70, is transported into the ER lumen. Its TMD assists in its retention in the ER, and eventually, the deposition of O10 inside PBs probably depends on the interaction with 16-kD γ-zein. Mutated o10 protein without the TMD may still be transported into the ER lumen with the aid of HIP because the O10 N terminus still can interact with HIP. Indeed, the results of subcellular localization in *N*. *benthamiana* leaves indicated that o10 co-localized with ER (Fig 4D). However, the dramatic decrease of o10 in the ER fraction suggested that the loss of TMD greatly affected the proper retention of o10 in the ER lumen. The o10 in ER might be degraded afterwards.

**Fig 8:** Model depicting the function of O10. In the wild-type kernel, O10 was first synthesized in the cytoplasm; HIP and HSP70 may have offered assistance when O10 was transported into the ER lumen. The TMD of O10 assisted with its retention in the ER. Finally, O10 was deposited in the interior of PB mainly depending on the aid of 16-kD γ-zein. In PB, O10 might determine the ring-shaped distribution of 16-kD γ-zein and 22-kD α-zein at the interface between the α-zein-rich core and the γ-zein-rich periphery of PB. The ring-shaped structure of 16-kD γ-zein and 22-kD α-zein is essential for maintaining the morphology of PB. In the o10 kernel, o10 was also transported inside the ER lumen, but it could not anchor onto the ER membrane as a result of the transmembrane deletion; thus, it might be degraded but not deposited in PB. This could affect the normal zein assembly, especially the 16-kD γ-zein and 22-kD α-zein, generating the misshapen PBs.

RETRACTED

### O10 affects the morphology of PBs by determining the distribution of 16-kD γ-zein and 22-kD α-zein

Previous studies found that the distribution of different zeins in PB showed restricted patterns. In general, the β- and γ-zeins were located in the periphery of PBs, while the α- and δ-zeins were located in the core of PB [12]. The mechanism for the special distribution of zeins is poorly understood. It was believed that the intrinsic hydrophilic-hydrophobic properties of different zeins and the direct interactions between them determined their proper distribution in PBs [44,45]. Further analysis revealed the distinct distributions of different α-zeins in PB. The 19-kD α-zein is located throughout the core of PB. However, the 22-kD α-zein has a special localization at the interface region between the α-zein-rich core and the γ-zein-rich periphery of PB [14]. In this study, we found that different γ-zeins also had distinct distributions. The 27-kD γ-zein and the 50-kD γ-zein were located throughout the peripheral region of PB. However, the 16-kD γ-zein, similar to the 22-kD α-zein, was also located at the interface between the core and the periphery of PBs (Fig 6). The specialized distribution of 22-kD α-zein and 16-kD γ-zein could not be fully explained by either their hydrophilic/hydrophobic properties or their interactions with other zeins. O10 could interact with both 22-kD α-zein and 16-kD γ-zein and co-localized with them (Fig 5). A loss of function of O10 would disrupt the ring-shaped distribution of 22-kD α-zein and 16-kD γ-zein (Fig 6). This suggested that O10 may be functionally responsible for the ring-shaped distribution of 22-kD α-zein and 16-kD γ-zein. Therefore, these three proteins form a newly defined structural zone of maize PBs, i.e., the ring-shaped interface region.

The ring-shaped interface was important for the morphology of PBs. The disruption of this interface region in *o10* may have led to the formation of misshapen PBs There is further evidence that the zein component of this interface region, namely the 22-kD α-zein and 16-kD γ-zein, are important for PB morphology. For example, an RNAi experiment in which the 22-kD α-zein alone was reduced caused misshapen PBs [46]. However, the reduction of both 19- and 22-kD α-zeins only severely restricted PB expansion but did not affect PB morphology [47]. These data suggested that the 22-kD α-zein might have a structural role in PB morphology. A frame-shift mutation of 16-kD γ-zein in *Mc1* led to angular PBs, suggesting that the 16-kD γ-zein might be functionally related to PB morphology [22,33]. The formation of this interface layer consisting of both α- and γ-zeins that was attached by non-zein protein O10 might function as an insulator for the hydrophilic peripheral region and the hydrophobic inner core of PB, thereby stabilizing the overall PB structure (Fig 8).

RETRACTED

Two opaque mutants, *o1* and *fl1*, share common features with *o10*. All three mutants have very minor changes in zein contents [14,23]. *o1* and *o10* endosperm both display misshapen PBs. Although O1 and O10 do not directly interact, they share a common potential interacting protein, namely HIP [23]. The accumulation of O10 significantly decreased in *o1*, which provided an explanation for the misshapen PBs in *o1* endosperm. FL1 could directly interact with α-zeins, and in *fl1*, the ring-shaped distribution of 22-kD α-zein was affected [14]. Since FL1 localizes in the PB membrane and 22-kD α-zein is deposited inside PBs away from the PB membrane, therefore previous researches have speculated that maybe some unidentified factors are involved in 22-kD α-zein targeting in addition to FL1 [14]. In this study, we found that FL1 could directly interact with O10 in tobacco cells (Fig 7) and the distribution of 22-kD α-zein was also affected in *o10*. This suggested a functional link between O10 and FL1 in determining the ring-shaped distribution of 22-kD α-zein. According to the above analysis, we speculated that O10 might firstly interact with 16-kD γ-zein in ER lumen. FL1 perhaps promotes 22-kD α-zein’s interaction with O10 near the PB membrane when O10 and 16-kD γ-zein are entering the PB (Fig 8). Then the complex consisting of O10, 16-kD γ-zein and 22-kD α-zein is targeted to the interface region between the α-zein-rich core and the γ-zein-rich periphery of PB, by some unknown mechanism. The functional relationship among O1, O10 and FL1 requires further investigation.

## Materials and Methods

### Plant materials

The maize *o10-N1356* stock was obtained from the Maize Genetics Cooperation stock center. The mutant was crossed into a W22 genetic background to produce the F2 populations. Kernels of the F2 ears exhibited a 3:1 segregation of wild-type kernels (*o10*/+ or +/+) and homozygous mutant kernels (*o10*/*o10*) were used for analysis. The root, stem, third leave, silk, tassel, and ear tissues were collected from at least three W22 plants at the V12 stage. The seeds were used for genetic transformation as in [17]. All of the plants were cultivated in a field at the Shanghai University campus in Shanghai, China.

### Measurement of protein, lipids and starch

For the protein measurements, the endosperm of *o10* and wild-type mature kernels was separated from the embryo and pericarp by dissection after soaking the kernels in water. The samples were dried to constant weight, pulverized with a mortar and pestle in liquid N_2_, and then measured according to a previously described protocol [17]. All of the measurements were replicated at least three times.

RETRACTED

For the lipid measurements, fifty mature kernels of the wild-type or *o10* were collected from well-filled, mature ears. The kernels were pulverized with a mortar and pestle in liquid N_2_, and 100 mg of dried flour was used for lipid extraction and then measured according to a previously described protocol [17]. All of the measurements were replicated at least three times.

For the starch measurements, fifty mature kernels of the wild-type and *o10* were ground in liquid N_2_. The resulting powders were dried to a constant weight. Finally, the total starch was measured using an amyloglucosidase/α-amylase starch assay kit (Megazyme). The protocol referenced the method in [20]. All of the measurements were replicated at least three times.

### Scanning electron microscopy and transmission electron microscopy

For scanning electron microscopy, the *o10* and wild-type mature kernels from the same F2 ear were prepared according to the previously described method [20]. The samples were observed with a scanning electron microscope (S3400N; Hitachi).

For transmission electron microscopy, immature kernels (21 DAP) of *o10* and the wild-type were prepared as previously described [17]. The samples were observed with a Hitachi H7600 transmission electron microscope.

### Map-based cloning

A population of 12,000 homozygous opaque kernels and 1500 wild-type kernels from F2 ears was used for gene mapping. Molecular markers that were distributed throughout maize (*Zea mays*) chromosome 1 were used for preliminary mapping. Molecular markers for fine mapping (S1 Table) were developed to localize the *o10* locus to a 110-kb region. The corresponding DNA fragments were amplified from *o10* and wild-type plants using KOD Plus DNA polymerase (Toyobo) and sequenced using a MegaBACE 4500 DNA analysis system (Amersham Biosciences).

### Polyclonal antibodies

Two O10 antibodies were produced in this study: anti-O10 and anti-O10-C. For anti-O10 antibody production, the cDNA sequence encoding the N terminus of O10 (1 aa–541 aa) was inserted into pGEX-4T-1 (Amersham Biosciences) at the *EcoRI-* and *BamHI*-digested sites. The primers were 5’-AAAAGAATTCATGGGCATGAGCTTGCACGCCGCGCG-3’ and 5’-CGCGGATCCTCATGATCCCACTGATTCAGCTAGAG-3’. The GST-tagged O10 fusion protein was purified using the ÄKTA protein purification system (GE Healthcare) with a GSTrap FF column. For anti-O10-C, the C-terminal peptides of O10 (1020 aa–1059 aa) were synthesized at Shanghai ImmunoGen Biological Technology. Both antibodies were prepared by Shanghai ImmunoGen Biological Technology in rabbits according to standard protocols.

RETRACTED

For 16-kD γ-zein, 19-kD α-zein, 22-kD α-zein, 27-kD γ-zein and 50-kD γ-zein antibody production, regions of low similarity of 16-kD γ-zein, 19-kD α-zein, 22-kD α-zein, 27-kD γ-zein and 50-kD γ-zein were selected according to a previous study [48]. The cDNAs responsible for the selected polypeptides were cloned into pGEX-4T-1 (Amersham Biosciences), and glutathione S-transferase-tagged fusion protein was purified with the ÄKTA purification system (GE Healthcare) using a GSTrap FF column. Antibodies were prepared by Shanghai ImmunoGen Biological Technology in rabbits according to standard protocols.

### The construction of transgene vectors and their transformation

For functional complementation transgene tests, a 3180-bp ORF sequence of *O10* with two restriction enzyme sites for *BamHI* and *SalI* was cloned by PCR using the following primers: 5’-CGCGGATCCATGGGCATGAGCTTGCACGCCGCGCG-3’ and 5’-CCGCTCGAGTCAGGGACGTTTTCTCTGCCCA-3’. The resulting fragment was cloned into a pHB vector, which carries a *bar* resistance marker and a CaMV 35S promoter. The CaMV 35S promoter was substituted by a 2 kb upstream DNA sequence from the start codon of *O10* with two restriction enzyme sites for *EcoRI* and *BamHI* for identical *O10* expression. The amplification primers were 5’-CCGGAATTCTCTGCTGCTGATGTCTTGT-3’ and 5’-GCGGATCCGGCCGTGTGCCGTAGTTT-3’. The construct was transferred into *Agrobacterium tumefaciens* (GV3101). *Agrobacterium*-mediated maize transformation was performed according to known protocols [49]. Five independent transgenic lines were generated. The transgenic lines were all backcrossed to *o10/o10* plants by two successive generations to obtain kernels with a homozygous *o10* locus. The SSR217401-a marker that was linked tightly with the *o10* locus was used to identify homozygous *o10* kernels.

To generate the RNAi construct, we used the fragment containing 384 bp from the cDNA of *O10* (30 bp-414 bp) according to the sequence analysis on http://rnaidesigner.thermofisher.com/rnaiexpress/. The forward-oriented fragment was amplified with the following pair of primers: 5’-CTTCTCGAGGCACGAGGATCTGAGCTG-3’ and 5’-CTTCCATGGTTTTCCACTACTTCTACCGA-3’ with restriction enzyme sites for *XhoI*/*NcoI*. The reverse fragment was amplified with the primers 5’-CTTTCTAGAGCACGAGGATCTGAGCTG-3’ and 5’-CTTGGATCCTTTTCCACTACTTCTACCGA-3’ with restriction enzyme sites for *XbaI*/*BamHI*. The construct was transferred into *Agrobacterium tumefaciens* (GV3101). *Agrobacterium*-mediated maize transformation was performed according to published protocols [49]. Six independent transgenic lines were generated. The transgenic lines were all backcrossed with W22 for 3 generations.

RETRACTED

### RNA extraction and real-time PCR analysis

For RNA extraction and Real-Time PCR analysis, the protocol referenced the method in [23]. The primers that were used for Real-Time PCR analysis are listed in S1 Table.

### Gel filtration chromatography

The total kernel protein (21 DAP) was extracted by grinding in liquid nitrogen and suspending in extraction buffer (50 mM Tris-Cl, 2.5 mM EDTA, 150 mM NaCl, 0.2% NP-40, 20% glycerol, 1 mM PMSF and 1% plant cocktail [Sigma Aldrich]) on ice for 20 min. The lysate was then centrifuged at 12,000 rpm for 5 min, the pellet was discarded, and the lysate was centrifuged one more time. A Superdex 200 10/300 GL Column (GE Healthcare) was first equilibrated in protein extraction buffer with an ÄKTA purifier system (GE Healthcare) until the UV baseline was smooth. A 500-μl volume of maize kernel lysate was injected into the system, and the flow speed was adjusted to 0.5 ml per minute. After the first volume (6 ml) flowed through, consecutive fractions of 500 μl each were then collected. The protein complex was then concentrated by acetone and analyzed by immunoblotting.

### Subcellular localization of O10 in *N*. *benthamiana*

The ORF sequences of *O10* and *o10* were amplified by PCR using KOD plus polymerase (Toyobo) with the primers 5’-CACCATGGGCATGAGCTTGCACGCCGCGCG-3’ and 5’-TCAGGGACGTTTTCTCTGCCCAA-3’. Amplified fragments were subcloned into pENTR/D-TOPO with the Gateway TOPO cloning kit (Invitrogen) and sequenced. The right entry clone was introduced into a pB7WGY2 plant expression vector through an LR reaction of the Gateway system (Invitrogen) [50]. The well-established fluorescent protein marker mCherry-HDEL was used to label the ER [51]. The expression vectors were transformed into *Agrobacterium tumefaciens* strain GV3101. The agro-infiltration procedure was performed as previously described [52].

### Subcellular fractionation and immunoblot analysis

The subcellular fractions of endosperm cell were prepared as previously described [23,53]. To peel off the ER surrounding PB, the separated PB fraction was resuspended in Buffer B (10 mM Tris-HCl, pH 8.5, 10 mM KCl, 5 mM MgCl_2_, 1 mM DTT, and proteinase inhibitor cocktail), added to 5% Triton X-100 [Sigma-Aldrich], shaken at 4°C for 4 h, and then centrifuged at 10,000 g and 4°C for 20 min. Then, the pellets were resuspended in an equal volume of Buffer B. Immunoblot analyses were performed as previously described [14]. The purified anti-O10, anti-O10-C and 22-kD α-zein antibodies were used at 1/500, while the anti-tubulin antibody (Sigma-Aldrich) and anti-BIP antibody (Santa Cruz Biotechnology) were used at 1/1000.

RETRACTED

### Yeast two-hybrid assay

All of the O10 bait constructs were made in pGBKT7. For the O10-N bait, the cDNA sequence of the N terminus of O10 (O10-N, 1 aa-268 aa) was fused downstream from the GAL4 BD domain in pGBKT7 at the *EcoRI* and *BamHI* restriction sites. The primers were 5’-AAAAGAATTCATGGGCATGAGCTTGCACGCCGCGCG-3’ and 5’-CGCGGATCCTCATTTGCTTTCTGCTTCATCAGA-3’. The clones were sequenced to ensure that an in-frame fusion with the GAL4 DNA binding domain had been created and that there were no mutations that would cause amino acid substitutions. For the pGADT7-preys, all of the zein-coding regions were amplified with genomic DNA (zein genes do not have introns). The primers were designed to exclude the 5’ region encoding the signal peptide and to incorporate an *EcoRI* site at the 5’ end and a *BamHI* at the 3’ end for cloning into pGADT7, with the exception of the 3’ primer for the 16-kD γ-zein, which was designed with an *XhoI* site, and the 5’ primer for the 50-kD γ-zein, which was designed with a *NedI* site. The coding regions of the O1-Tail (877–1520 aa), FL1 and HIP were amplified with maize endosperm cDNA that carried restriction sites for *EcoRI*/*PstI*, *EcoRI*/*BamHI* and *SfiI*/*BamHI*, respectively. The primers that were used for amplification are listed in S1 Table. The zeins, O1-Tail, FL1, and HIP were cloned and inserted in-frame into pGADT7. Yeast strain AH109 was co-transferred with pGBKT7-O10-N and pGADT7-Preys. The interaction between T-antigen and Human P53 was used as a positive control. The interaction between pGBKT7-O10-N and pGADT7-empty was used as a negative control. The putative positive clones were further spotted with a dilution series onto SD/-Leu/-Trp medium and SD/-Ade/-His/-Leu/-Trp medium.

### LCI assay

To confirm the interaction between O10 and different types of zeins or HIP, the cDNA sequence of the N terminus of O10 (O10-N, 1–268 aa) was cloned into JW771 (NLUC), the full-length ORF of HIP, and all of the zein coding regions without the 5’ region encoding the signal peptide were cloned into JW772 (CLUC), yielding O10-N-NLUC and ZEIN/HIP-CLUC constructs for the LCI assay. To analyze the interaction between O10 and O1 or FL1, the full-length ORF of O10 was cloned into JW772 (CLUC), and the cDNA sequences of C terminus of O1 (877 aa-1520 aa) and FL1 (150 aa-302 aa) were cloned into JW771 (NLUC), yielding O10-CLUC and O1-C/FL1-C-NLUC constructs for the LCI assay.

The constructs were transformed into *Agrobacterium tumefaciens* strain GV3101. The agro-infiltration procedure was performed as previously described [50], and the resulting luciferase signals were captured using the Tanon-5200 image system. These experiments were repeated at least three times with similar results.

RETRACTED

### Immunolabeling

Immunolabeling was performed as previously described [20]. The purified anti-O10 antibody was used at 1/200; the 22-kD α-zein and 50-kD γ-zein antibodies were used at 1/1000; and the 16-kD γ-zein, 19-kD α-zein and 27-kD γ-zein antibodies were used at 1/5000.

### HPLC analysis of zeins

To measure the zeins, 10 wild-type and *o10* kernels were ground into powder in liquid N_2_, and 150 mg of dry powder was dissolved in 1 ml of extract buffer (70% ethanol, 5% β-mercaptoethanol, and 0.5 sodium acetate (w/v)). The samples were shaken at room temperature for at least 4 h and centrifuged at 500 g for 20 min at room temperature. The supernatants were diluted 5 times and measured by HPLC. The relative concentrations of the zeins were computed using their peak areas. All of the measurements were repeated three times.

### Accession numbers

Sequence data from this article can be found in the GenBank/EMBL data libraries under the following accession numbers: *10-kD δ-zein*, AF371266; *15-kD β-zein*, M12147 (GRMZM2G086294); *16-kD γ-zein*, AF371262 (GRMZM2G060429); *18-kD δ-zein*, AF371265 (GRMZM2G100018); *19-kD α-zein*, M12146 (AF546188.1); *22-kD α-zein*, NM_001112529 (GRMZM2G044625); *27-kD γ-zein*, AF371261 (GRMZM2G138727); *50-kD γ-zein*, BT062750 (GRMZM2G138689); *O1*, GRMZM2G449909; *FL1*, NM_001112594 (GRMZM2G094532); *O10*, XM_008667043.1 (GRMZM2G346263); Zm *HIP*, GRMZM2G023275; and Zm *UBQ*, BT018032.

## Supporting Information

S1 Fig Cytological observation and biochemical analysis of the wild-type and *o10* endosperm. (A) Scanning electron microscopy of the wild-type and *o10* endosperm. Bars = 20 μm. (B) Resin slice observation of the wild-type and *o10* endosperm at 12 DAP and 18 DAP. Bars = 50 μm. (C) SDS-PAGE analysis of the total protein extracts from the endosperm of developing wild-type and o10 kernels (18 DAP and 24 DAP) and mature kernels. (D) Protein quantification of total protein, zein and non-zein extracted from the endosperm of wild-type and *o10* mature kernels. (E) Comparison of the total starch content in the wild-type and *o10* mature kernels. (F) Comparison of the total lipid content in the wild-type and *o10* mature kernels.
(PDF)

S2 Fig Phenotyping and genotyping of transgenic kernels, the expression of *O10* and the accumulation of O10 in RNAi lines. (A) The transgenic events (T0 lines) were hybridized to the homozygous mutant (*o10*/*o10*) and self-pollinated (T2 lines). Using the molecular marker linked to the *o10* locus, ten vitreous and ten opaque homozygous mutant kernels were sorted out from T2 ears. -, H_2_O control. (B) Light transmission and the transverse section of the ten vitreous and ten opaque homozygous mutant kernels were observed. Bars = 1 cm. (C) Using the primers of the *bar* gene to identify the transgenic negative and positive kernels. +, *PHB* vector. (D) The RNAi transgenic events (T0 lines) were hybridized to the W22 background and then self-pollinated (T2 lines), underwent light transmission and used to take transverse sections of the vitreous and opaque kernels from T2 ears. Bars = 1 cm. (E) Using the primers of the *bar* gene to identify the transgenic negative and positive kernels. +, *pFGC5941* vector. (F) Real-time quantitative PCR was used to analyze the RNA expression of *O10* at 21 DAP in the transgenic negative (RNAi (+)) and positive (RNAi (-)) mature kernels. An immunoblot analysis was performed to compare the accumulation of O10 in the transgenic negative and positive mature kernels. Anti-tubulin was used as a sample loading control.
(PDF)

S3 Fig Sequence alignment of the proteins. (A) Sequence alignment of seven O10 repeats and the homologous sequence in other cereal species. (B) Sequence alignment of the transmembrane domain of O10 and its homologous sequence in other species.
(PDF)

S4 Fig Immunoblots and SDS-PAGE were used to analyze the molecular weight of O10. (A) Immunoblot analysis of O10 in separated proteins with anti-O10 antibody. The total protein of maize kernel (21 DAP) was separated into 10 parts by gel filtration chromatography. The bands of 43 kD, 75 kD, 158 kD and 440 kD were the gel filtration markers. (B) Immunoblot analysis of the O10 molecular weight by adding different denaturants and reducing agents before the thermal denaturation of samples. Panel 1, 10% (W/V) SDS; Panel 2, 10% (W/V) SDS + 100 mM DTT; Panel 3, 10% (W/V) SDS + 5% (V/V) β-Mercaptoethanol; Panel 4, 10% (W/V) SDS + 8 M urea.
(PDF)

S5 Fig Kyte-Doolittle Hydropathy Analysis of the seven-repeat domain of O10. The hydropathy characteristics of the seven-repeat domain of O10 were determined by the method of Kyte and Doolittle (http://ca.expasy.org/tools/protscale.html).
(PDF)

S6 Fig The expression of *O10* in the wild-type and mutant kernels during maize kernel development. Ubiquitin was used as the internal control.
(PDF)

S7 Fig RNA expression analysis of different zein genes during maize kernel development. (A) The expression of *10-kD δ-zein* in the wild-type and mutant kernels at 18DAP and 24DAP. (B) The expression of *15-kD β-zein* in the wild-type and mutant kernels at 18DAP and 24DAP. (C) The expression of *16-kD γ-zein* in the wild-type and mutant kernels at 18DAP and 24DAP. (D) The expression of *19-kD α-zein* in the wild-type and mutant kernels at 18DAP and 24DAP. (E) The expression of *22-kD α-zein* in the wild-type and mutant kernels at 18DAP and 24DAP. (F) The expression of *27-kD γ-zein* in the wild-type and mutant kernels at 18DAP and 24DAP. (G) The expression of *50-kD γ-zein* in the wild-type and mutant kernels at 18DAP and 24DAP. Ubiquitin was used as the internal control. For each sample, three technical and two independent biological replicates were performed. The values are the mean values with SE (n = three individuals; ***P<0.001, Student’s *t* test).
(PDF)

S8 Fig HPLC analysis of the content of 16-kD γ-zein in the wild-type and *o10* mature kernels. (A) The peak diagram of HPLC from the determination of the zein content in mature kernels of the wild-type and *o10*. (B) The relative concentrations of 16-kD γ-zein in the wild-type and *o10* mature kernels.
(PDF)

S1 Table The primers used in this study. (PDF)
